The article "Retrospective Analysis of the Clinical Efficacy of Early Goal-Directed Therapy Combined with Meticulous Nursing Intervention in Patients with Posttraumatic Sepsis" was published in 2021. Journal: J Healthc Eng.

# Retrospective Analysis of the Clinical Efficacy of Early Goal-Directed Therapy Combined with Meticulous Nursing Intervention in Patients with Posttraumatic Sepsis

**DOI:** 10.1155/2021/6706464

**Published:** 2021-12-13

**Authors:** Zhe Yuan, Shilu Yang, Chunhua Zhang, Ke Chen, Minhuan Wang, Shaoqian Hao, Shimin Dong, Yang Yang

**Affiliations:** ^1^Department of Emergency, The Third Hospital of Hebei Medical University, Shijiazhuang 050051, Hebei, China; ^2^Department of Care Unit, Wuhan Jinyintan Hospital, Wuhan 430011, Hubei, China; ^3^Department of Cardiology, The Third Hospital of Hebei Medical University, Shijiazhuang 050051, Hebei, China

## Abstract

**Objective:**

To explore the intervention effect of early goal-directed therapy (EGDT) combined with meticulous nursing on patients with posttraumatic sepsis.

**Methods:**

The data of 50 patients with posttraumatic sepsis undergoing EGDT in the emergency department of our hospital from January 2020 to December 2020 were retrospectively analyzed. According to different nursing methods, they were divided into control group (*n* = 25) with routine nursing measures and observation group (*n* = 25) with meticulous nursing measures. The application effect of the two nursing modes was scientifically evaluated.

**Results:**

No statistical differences in general data were found between the two groups (*P* > 0.05). After 6 h of intervention, the circulatory function, oxygenation function, and renal function of both groups were better than those before intervention, and central venous pressure (CVP), mean arterial pressure (MAP), blood oxygen (PaO_2_), oxygenation index (PaO_2_/FiO_2_), central venous oxygen saturation (ScvO_2_), and urine volume in the observation group were notably higher than those in the control group (*P* < 0.05). The heart rate (HR), serum creatinine (SCr), and blood lactic acid in the observation group were notably lower than those in the control group (*P* < 0.05). The 28-day survival rate and quality of life after intervention in the observation group were notably higher than those in the control group, with obvious differences between the two groups (*P* < 0.05).

**Conclusion:**

Meticulous nursing intervention for patients with posttraumatic sepsis undergoing EGDT can effectively improve the body's functional indexes, which is superior to the routine nursing in controlling the patients' condition, improving the survival rate and quality of life after intervention, and ensuring the clinical treatment effect. Therefore, it is worthy of promotion.

## 1. Introduction

Although progress has been made in the treatment of primary injuries after severe trauma, the incidence and mortality of posttraumatic sepsis have not been controlled well [1–4]. According to statistics, infection, second only to shock, is one of the main causes of sepsis and death after trauma, which can lead to multiple organ dysfunction syndrome (MODS) and even death in severe cases if not properly treated [3, 5–7]. Early goal-directed therapy (EGDT) can improve the condition and prognosis of patients with sepsis, and clinical nursing is a key link to ensure the continuity of treatment, with an extremely important role. However, there are few studies on monitoring the nursing effect of patients with sepsis undergoing EGDT in China, especially on monitoring the nursing effect on those with posttraumatic sepsis. Based on this, this study focused on comparing the effect of EGDT combined with meticulous nursing or routine nursing on circulatory function, oxygenation function, renal function, blood lactic acid, and survival rate of patients. Fifty patients with posttraumatic sepsis undergoing EGDT in the emergency department of our hospital from January 2020 to December 2020 were selected and grouped according to different nursing methods to conduct a retrospective study, aiming to seek nursing methods to promote the rehabilitation and improve the nursing cooperation of patients.

The article "Retrospective Analysis of the Clinical Efficacy of Early Goal-Directed Therapy Combined with Meticulous Nursing Intervention in Patients with Posttraumatic Sepsis" was published in 2021. Journal: J Healthc Eng.

## 2. Study Protocol

### 2.1. Objects

Referring to *2016 International Guidelines for Management of Sepsis and Septic Shock* [8], the enrolled patients (≥18 years old) met at least two of the following diagnostic criteria: (1) body temperature >38 °C or < 36 °C; (2) heart rate >90 times/min; (3) respiratory rate >20 times/min or partial pressure of carbon dioxide (PCO_2_) < 4.25Kpa/32 mmHg; and (4) white blood cell count >12 × 10^9^/L or < 4 × 10^9^/L, or immature neutrophils >10%. The following patients were excluded: (1) patients with hospitalization time less than 24 h; (2) patients who gave up treatment; (3) patients with autoimmune diseases, immunodeficiency diseases, and tumors; (4) patients who received immunosuppressive therapy recently; (5) patients who had infectious diseases or took antibiotics within a week; (6) patients with chronic diseases or long-term medication; and (7) patients without posttraumatic sepsis. The data of 50 patients with posttraumatic sepsis undergoing EGDT from January 2020 to December 2020 were retrospectively analyzed.

### 2.2. Grouping

According to different nursing methods, the enrolled 50 patients were equally divided into the control group and the observation group. All patients underwent EGDT, and patients in the control group received routine nursing, while those in the observation group received meticulous nursing. This study was approved by the Hospital Ethics Committee, and the family members of patients signed the informed consent.

The article "Retrospective Analysis of the Clinical Efficacy of Early Goal-Directed Therapy Combined with Meticulous Nursing Intervention in Patients with Posttraumatic Sepsis" was published in 2021. Journal: J Healthc Eng.

The flow diagram of the study is shown in Figure 1.

### 2.3. Methods

*EGDT*. After admission of the patients, the nursing staff should quickly establish the venous channels, provide sufficient blood volume, ensure tissue perfusion through gastrointestinal and venous supply, and rapidly expand the volume to increase cardiac oxygen-carrying capacity and blood output, thus ensuring the oxygen supply of body tissue, restoring circulating blood volume, shortening the time of insufficient blood perfusion, and avoiding multiple organ failure [9–12]. When establishing the venous channels, venous indwelling needles were selected to puncture the large blood vessels near the heart. Three venous channels were established: one for blood test, another for pumping special vasopressors such as dopamine, and the other for pumping a large number of drugs and liquids. For patients with insufficient blood volume, fluid supplements should be reasonably selected according to hemodynamics, central venous pressure, and hematocrit, with controlled infusion speed. Glucose liquid could be injected fast, while normal saline should be slow. Colloid and crystalloid solutions should be crossed to avoid heart failure and pulmonary edema. Continuous pumping of insulin promoted glucose metabolism and prevented hyperglycemia [7, 13–15].

The patients in the control group received routine nursing by closely observing the changes in vital signs (body temperature, heart rate, blood pressure, respiration, and oxygen saturation), oxygen inhalation, fluid infusion, accurately recording urine volume, and the 24-hour fluid intake and output, and implementing effective anti-infection measures according to doctor's advice to prevent complications [16].

The patients in the observation group received meticulous nursing, specifically as follows. (1) *Training*. The nursing staff were organized to learn sepsis-related knowledge and master hemostasis, arterial catheterization, collection of arterial blood gas, measurement of central venous pressure (CVP), and other skills [17]. (2) *Team Awareness*. Teamwork was emphasized, and the staff complemented each other's advantages to give full play to team advantages. (3) *Nursing Process*. ① At the 1st hour, the patients' condition was quickly assessed, and relevant departments were notified to control active bleeding of the open wound and effectively stop bleeding through compression hemostasis or use of compression tourniquet. The patients' consciousness, body temperature, heart rate, respiration, blood pressure, and oxygen saturation were closely monitored, and mechanical ventilation was applied if necessary. Three venous channels were quickly established, the catheter was indwelled in the vein with large diameter, and the central venous access was established as soon as possible. The patients were infused with heated transfusion, and the speed of fluid infusion was first fast and then slow. Blood was collected to determine the patients' blood loss, preoperative and pretransfusion preparations were made, and arterial blood gas was checked to quickly assess their condition. The catheter was retained, and precise urine bags were used to accurately record hourly urine volume of patients. ② At the 2nd hour, the patients' consciousness, heart rate, respiration, blood pressure, oxygen saturation, and urine volume were closely monitored. Their skin color (eyelids, lips, and nail bed), elasticity, and capillary filling time were dynamically assessed. With warm and pressurized blood transfusion, the bleeding of open wound was dynamically assessed. Temperature control blankets were applied to keep warm, dispel chills, and reduce oxygen consumption. The invasive blood pressure (ABP) was monitored by indwelling the catheter, and the infusion speed was adjusted according to ABP to maintain the mean arterial pressure (MAP) above 65 mmHg. Blood pressure should not be too high to prevent aggravating bleeding and excessive fluid load. ③ At the 3rd hour, the patients' consciousness, heart rate, respiration, blood pressure, oxygen saturation, and urine volume were closely monitored. Their skin color (eyelids, lips, and nail bed), elasticity, capillary filling time, and bleeding of open wound were dynamically assessed. Those with drainage tubes were assessed for drainage conditions such as volume, color, and character of drainage fluid. Vasoactive drugs were taken according to the doctor's advice, and two-channel pumps were adopted alternately to prevent blood pressure fluctuations. CVP and central venous oxygen saturation (ScvO_2_) were accurately measured to guide the speed of fluid infusion. Analgesia and sedation were performed, oxygen consumption was reduced to meet ScvO_2_ standard, and analgesic and sedative effect was dynamically assessed. ④ From the 4th hour to the 5th hour, the patients' consciousness, heart rate, respiration, blood pressure, oxygen saturation, and urine volume were closely monitored. Their skin color (eyelids, lips, and nail bed), elasticity, capillary filling time, and bleeding of open wound were dynamically assessed. Those with drainage tubes were assessed for drainage conditions such as volume, color, and character of drainage fluid. The analgesic and sedative effect was dynamically assessed, and the speed of fluid infusion and vasoactive drugs was adjusted according to ABP. ⑤ At the 6th hour, CVP and ScvO_2_ were measured to guide the infusion speed, and blood gas was reviewed. The above meticulous nursing intervention combined with EGDT for patients with posttraumatic sepsis could prevent complications such as infection, thrombosis, and multiple organ failure.

The article "Retrospective Analysis of the Clinical Efficacy of Early Goal-Directed Therapy Combined with Meticulous Nursing Intervention in Patients with Posttraumatic Sepsis" was published in 2021. Journal: J Healthc Eng.

### 2.4. Observation Indexes

The monitoring data of the two groups after 6 hours were observed. (1) Circulation function. The CVP and MAP levels of the patients were detected by automatic and noninvasive manometry, and the heart rate (HR) was measured at the same time. (2) Oxygenation function. The partial pressure of blood oxygen (PaO_2_), oxygenation index (PaO_2_/FiO_2_), and ScvO_2_ of patients were obtained through blood gas analysis. (3) Renal function. The urine volume and serum creatinine (SCr) were detected to further analyze the renal function of patients. (4) Blood lactic acid. Colorimetry was adopted to determine the plasma lactic acid levels of the two groups. (5) 28-day survival rate. Survival of the two groups within 28 days was recorded to calculate the survival rate. (6) Hospitalization time. The hospitalization time of the two groups was recorded. (7) Quality of life. The quality-of-life scale (SF-36) was used to evaluate the living conditions of patients after 1 month of intervention. The scale was a universal measurement scale developed by the American Medical Outcomes Study, which contained 36 items and involved role function, physical function, cognitive function, social function, and emotional function. The full score of each dimension was 100 points, and a higher score represented the higher quality of life.

### 2.5. Statistical Processing

The data in this study were processed by SPSS 22.0 software and graphed by GraphPad Prism 7 (GraphPad Software, San Diego, USA). The data included enumeration data and measurement data, which were expressed as (n (%)) and (‾*x* ± *s*), and tested by chi-square and *t*-test. The differences were considered statistically different when *P* < 0.05.

## 3. Results

### 3.1. General Information

No statistical differences in age, gender, APACHE II score, LAC, infection sites, infection types, and underlying diseases were found between the two groups (*P* > 0.05), which were suitable for control study, as shown in Table 1.

### 3.2. Circulatory Function

After 6h of intervention, the indexes of circulatory function in both groups were better than those before intervention, and CVP and MAP in the observation group were notably higher than those in the control group (*P* < 0.05), with notably lower HR in the observation group than that in the control group (*P* < 0.05), as shown in Table 2.

The article "Retrospective Analysis of the Clinical Efficacy of Early Goal-Directed Therapy Combined with Meticulous Nursing Intervention in Patients with Posttraumatic Sepsis" was published in 2021. Journal: J Healthc Eng.

### 3.3. Oxygenation Function

After intervention, the indexes of oxygenation function in both groups notably increased, and the indexes in the observation group were obviously higher than those in the control group (*P* < 0.05), with statistical value, as shown in Table 3.

### 3.4. Renal Function

The urine volume in both groups increased after intervention, and the volume in the observation group was higher than that in the control group (*P* < 0.05); SCr in both groups decreased after intervention, and SCr in the observation group was notably lower than that in the control group (*P* < 0.05), with statistically significant differences between the two groups, as shown in Table 4.

### 3.5. Blood Lactic Acid

After 6h of intervention, the blood lactic acid levels of both groups decreased, and the level in the observation group was notably lower than that in the control group (*P* < 0.05), with statistical significance, as shown in Figure 2.

### 3.6. 28-Day Survival Rates and Hospitalization Time

The 28-day survival rate in the observation group was notably higher than that in the control group (*P* < 0.05), while the hospitalization time in the observation group was notably shorter than that in the control group (*P* < 0.05), with statistical value, as shown in Table 5.

### 3.7. Quality of Life

The quality-of-life indexes (role function, cognitive function, physical function, emotional function, and social function) in the observation group were notably better than those in the control group (*P* < 0.05), with statistical significance, as shown in Table 6.

## 4. Discussion

After severe trauma such as multiple injuries, craniocerebral injury, hemorrhagic shock, burn, fractures, and large surgical wound, poor blood perfusion causes ischemia, hypoxia, wound infection, stress response, and gastrointestinal paralysis, thus easily leading to a series of pathological symptoms such as infection and systemic inflammatory response syndrome (SIRS) complicated with sepsis, septic shock, MODS, and even death [18–21]. At present, many measures related to EGDT and cluster therapy have been formed according to the sepsis treatment guidelines in clinical practice. EGDT helps to improve the cognition of clinicians on posttraumatic sepsis and has gradually become a routine measure for the treatment of sepsis due to its excellent clinical application effect. However, in recent years, many scholars have put forward the importance of nursing intervention in EGDT from different perspectives and believe that routine nursing can easily ignore individual differences. In addition, HSU et al [22] have stated in their report that meticulous nursing mode can effectively prevent further deterioration of sepsis and play an important role in reducing its mortality. Based on the above background, this study actively explored the intervention effect of EGDT combined with meticulous nursing or routine nursing on patients with posttraumatic sepsis, aiming to explore long-term and effective clinical nursing schemes.

The article "Retrospective Analysis of the Clinical Efficacy of Early Goal-Directed Therapy Combined with Meticulous Nursing Intervention in Patients with Posttraumatic Sepsis" was published in 2021. Journal: J Healthc Eng.

The results showed that after 6h of intervention, the circulatory function, oxygenation function, and renal function of both groups were better than those before intervention, and CVP, MAP, PaO_2_, PaO_2_/FiO_2_, ScvO_2_, and urine volume in the observation group were notably higher than those in the control group (*P* < 0.05); HR, SCr, and blood lactic acid in the observation group were notably lower than those in the control group (*P* < 0.05), which was consistent with the research results of Kleinpell et al [23]. This is enough to show that the circulation function, oxygenation function, and renal function of the observation group after intervention were better than those of the control group, and the related indexes of the observation group were closer to the normal levels. The meticulous nursing model implemented in the observation group is guided by holistic nursing, based on evidence-based nursing and patient-oriented, which focuses on the control of nursing quality. Compared with routine nursing, this nursing process pays more attention to nursing details to make the nursing work more effective, reasonable, and controllable, thereby greatly improving the body function of patients and effectively reducing organ injury. In addition, the 28-day survival rate and quality of life after intervention in the observation group were notably higher than those in the control group (*P* < 0.05), further confirming the intervention effect of meticulous nursing in EGDT. Meticulous nursing is superior to routine nursing in promoting the rapid rehabilitation of patients, greatly shortening their hospitalization time, and improving the survival rate and quality of life, which is an effective intervention measure to ensure the therapeutic effect of patients.

The study also has some shortcomings. Nursing measures in this study were developed based on EGDT in patients with posttraumatic sepsis, and the application effect of meticulous nursing was confirmed. However, the nursing measures only involved 6 hours, so the long-term intervention mechanism of meticulous nursing remains to be further explored. In addition, this study has a small sample size. To reduce the deviation in medical research and clinical practice, the sample size should be expanded to further confirm the application effect of meticulous nursing. In summary, the research flow should be designed in advance in the subsequent relevant studies to predict the relevant outcomes, and the sample size should be maximally extended to guarantee the accuracy of the results. In addition, more research dimensions should be studied as well.

The article "Retrospective Analysis of the Clinical Efficacy of Early Goal-Directed Therapy Combined with Meticulous Nursing Intervention in Patients with Posttraumatic Sepsis" was published in 2021. Journal: J Healthc Eng.

## 5. Conclusion

In conclusion, the observation group achieved significantly better indexes such as circulatory function, oxygenation function, renal function, blood lactic acid, and survival rate compared with the control group. This shows that meticulous nursing intervention for patients with posttraumatic sepsis undergoing EGDT can effectively improve the body's functional indexes, which is superior to the routine nursing in controlling the patients' condition, improving the survival rate and quality of life after intervention, and ensuring the clinical treatment effect. Therefore, it is worthy of promotion.

## Figures and Tables

**Figure 1:** Flow diagram of the study.

**Figure 2:** Comparison of blood lactic acid levels between the two groups (‾*x* ± *s*). Note: the abscissa represents before and after intervention, and the ordinate intervention represents the blood lactic acid level (mmol/L). The blood lactic acid levels in the control group before and after intervention were 7.2 ± 2.7 and 5.8 ± 2.5, respectively. The blood lactic acid levels in the observation group before and after intervention were 6.9 ± 2.6 and 4.3 ± 1.8, respectively. ^*∗*^ indicates an obvious difference in the blood lactic acid levels between the two groups after intervention (*t* = 2.4346, *P*=0.0187).

**Table 1:** Comparison of general data between the two groups (*n* = 25).

Indexes	Control group	Observation group	X^2^/*t*	*P*
Age (years)	48.72 ± 4.89	49.15 ± 4.93	0.3096	0.7582
Gender				
Male	17(68%)	18(72%)	0.0952	0.758
Female	8(32%)	7(28%)		
APACHE II score	17.92 ± 5.61	18.27 ± 5.58	0.2212	0.8259
Lac (mmol/L)	5.79 ± 1.63	5.84 ± 1.93	0.0990	0.9216
Infection sites				
Lungs	15(60%)	17(68%)	0.3472	0.556
Abdomen	5(20%)	3(12%)	0.5952	0.440
Urinary system	2(8%)	1(4%)	0.3546	0.552
Nervous centralis	1(4%)	3(12%)	1.0870	0.297
Others	4(16%)	3(12%)	0.1661	0.684
Infection types				
Bacterial infection	13(52%)	16(64%)	0.7389	0.390
Mycotic infection	4(16%)	2(8%)	0.7576	0.384
Underlying diseases				
Diabetes	8(32%)	9(36%)	0.0891	0.765
Coronary heart disease	10(40%)	7(28%)	0.8021	0.370
Chronic obstructive pulmonary disease	6(24%)	8(32%)	0.3968	0.529
Chronic liver disease	2(8%)	1(4%)	0.3546	0.552

**Table 2:** Comparison of indexes of circulatory function between the two groups (‾*x* ± *s*).

Group	CVP (cmH_2_O)		MAP (mmHg)		HR (times/min)	
	Before intervention	6h after intervention	Before intervention	6h after intervention	Before intervention	6h after intervention
Control group	3.4 ± 1.8	7.5 ± 2.3	62.2 ± 6.1	68.3 ± 5.8	129.1 ± 10.3	103.6 ± 5.1
Observation group	3.3 ± 1.7	10.9 ± 2.5	61.7 ± 5.9	81.6 ± 6.2	128.8 ± 10.4	90.5 ± 6.0
t	5.0043		7.8327		8.3178	
*P*	<0.0001		<0.0001		<0.0001	

The article "Retrospective Analysis of the Clinical Efficacy of Early Goal-Directed Therapy Combined with Meticulous Nursing Intervention in Patients with Posttraumatic Sepsis" was published in 2021. Journal: J Healthc Eng.

**Table 3:** Comparison of indexes of oxygenation function between the two groups (‾*x* ± *s*).

Group	PaO_2_ (mmHg)		PaO_2_/FiO_2_ (mmHg)		ScvO_2_ (%)	
	Before intervention	6h after intervention	Before intervention	6h after intervention	Before intervention	6h after intervention
Control group	100.1 ± 23.2	106.5 ± 24.4	238.4 ± 43.7	331.2 ± 33.3	56.2 ± 6.4	66.4 ± 4.3
Observation group	100.6 ± 24.1	145.7 ± 21.5	239.1 ± 44.1	364.1 ± 38.5	56.8 ± 6.6	77.1 ± 3.9
*t*	6.0269		3.2316		9.2159	
*P*	<0.0001		0.0022		<0.0001	

**Table 4:** Comparison of indexes of renal function between the two groups (‾*x* ± *s*).

Group	Urine volume (ml/h)		SCr (*μ*mol/L)	
	Before intervention	After intervention	Before intervention	After intervention
Control group	22.7 ± 10.8	38.2 ± 13.1	138.7 ± 20.1	126.1 ± 14.3
Observation group	22.5 ± 10.6	69.5 ± 11.6	138.9 ± 19.8	113.5 ± 15.2
*t*	8.9440		3.0188	
*P*	<0.001		0.0041	

**Table 5:** Comparison of 28-day survival rates and hospitalization time between the two groups.

Group	*n*	28-day survival rate (%)	Hospitalization time (d)
Control group	25	11(44)	17.04 ± 2.75
Observation group	25	18(72)	14.06 ± 2.87
t/*X*^2^		4.0230	3.7486
*P*		0.045	0.0005

**Table 6:** Comparison of SF-36 scores between the two groups (‾*x* ± *s*).

Dimensions	Control group	Observation group	*t*	*P*
Role function	72.01 ± 3.16	88.27 ± 4.28	15.2815	<0.0001
Cognitive function	70.94 ± 5.47	90.01 ± 4.65	13.2811	<0.0001
Physical function	73.04 ± 4.38	89.11 ± 5.69	11.1899	<0.0001
Emotional function	72.89 ± 3.41	89.27 ± 5.70	12.3004	<0.0001
Social function	76.15 ± 4.93	93.52 ± 2.84	15.2649	<0.0001

## Data Availability

The datasets used and/or analyzed during this study are available from the corresponding author on reasonable request.
